The article "IL-1β/HMGB1 signalling promotes the inflammatory cytokines release via TLR signalling in human intervertebral disc cells" was retracted in 2026. Reasons: manipulated data; manipulated images; plagiarized data; overlap with other authors' work.

# IL-1β/HMGB1 signalling promotes the inflammatory cytokines release via TLR signalling in human intervertebral disc cells

**DOI:** 10.1042/BSR20160118

**Published:** 2016-09-16

**Authors:** Fang Fang, Dianming Jiang

**Affiliations:** * Department of Orthopaedics, the First Affiliated Hospital of Chongqing Medical University, 400016, Chongqing, China

**Keywords:** high mobility group box 1 (HMGB1), interleukin (IL)β, intervertebral disc degeneration (IDD)

## Abstract

Inflammation and cytokines have been recognized to correlate with intervertebral disc (IVD) degeneration (IDD), via mediating the development of clinical signs and symptoms. However, the regulation mechanism remains unclear. We aimed at investigating the regulatory role of interleukin (IL)β and high mobility group box 1 (HMGB1) in the inflammatory response in human IVD cells, and then explored the signalling pathways mediating such regulatory effect. Firstly, the promotion to inflammatory cytokines in IVD cells was examined with ELISA method. And then western blot and real time quantitative PCR were performed to analyse the expression of toll-like receptors (TLRs), receptors for advanced glycation endproducts (RAGE) and NF-κB signalling markers in the IL-1β- or (and) HMGB1-treated IVD cells. Results demonstrated that either IL-1β or HMGB1 promoted the release of the inflammatory cytokines such as prostaglandin E2 (PGE2), TNF-α, IL-6 and IL-8 in human IVD cells. And the expression of matrix metalloproteinases (MMPs) such as MMP-1, -3 and -9 was also additively up-regulated by IL-1β and HMGB1. We also found such additive promotion to the expression of TLR-2, TLR-4 and RAGE, and the NF-κB signalling in intervertebral disc cells. In summary, our study demonstrated that IL-1β and HMGB1 additively promotes the release of inflammatory cytokines and the expression of MMPs in human IVD cells. The TLRs and RAGE and the NF-κB signalling were also additively promoted by IL-1β and HMGB1. Our study implied that the additive promotion by IL-1β and HMGB1 to inflammatory cytokines and MMPs might aggravate the progression of IDD.

## INTRODUCTION

Intervertebral disc (IVD) degeneration (IDD) is clinically characteristic of chronic low back pain and the secondary symptoms and signs of disc herniation, spinal canal stenosis and spinal deformities [1]. And such spinal disorders lead the disability causes of in the workforce [2]. The aetiology of IDD is complicated with multiple factors such as aging, sustained stress, heredity, smoking, obesity and trauma [3–5]. However, the molecular mechanisms underlying IDD are largely unknown. IDD is mainly characterized in pathology of reduced (and abnormal) intervertebral disc cells, of broken-down extracellular matrix (ECM), and of promoted pro-inflammatory mediators [6,7], which then progressively cause IDD damage in structure and function. Matrix metalloproteinase (MMP) is widely considered to play a role in disc degeneration by degrading collagen and proteoglycans found in the matrix [8–10]. Studies reported that MMP expression was associated with the degradation of the matrix in IDD. However, the regulation on the MMP expression was not clear.

The article "IL-1β/HMGB1 signalling promotes the inflammatory cytokines release via TLR signalling in human intervertebral disc cells" was retracted in 2026. Reasons: manipulated data; manipulated images; plagiarized data; overlap with other authors' work.

Interleukin (IL)-1 family is a group of cytokines (11 members), which is a key regulator in immune and inflammatory responses to infections or sterile insults [11,12]. The proinflammatory IL-1β is the most important cytokine, with a strong stimulation to the production of multiple proinflammatory mediators such as cytokines, chemokines and MMPs [12–14]. IL-1β expression has been reported to be significantly promoted in IDD tissues and cells [15], exerting regulation in multiple pathological processes of disc degeneration [16]. On the other side, the inhibition of IL-1β has been observed to promote ECM repair and block disc degeneration [17,18].

High mobility group box 1 (HMGB1) is DNA-binding chromatin protein. Nuclear HMGB1 organizes DNA and regulates gene transcription [19], via interacting with nucleosomes, transcription factors and histones [20]. The nucleus-resided HMGB1 has been observed to be released to cytosol and even extracellular space upon inflammatory and other stimulation [21,22] to mediate inflammation in multiple injury models [23–25]. Recently, HMGB1 has been recognized as a potent proinflammatory mediator in degenerated human discs [26]. And it was markedly up-regulated in the IVD in a lipopolysaccharide (LPS)-induced rat IDD model [27]. Toll-like receptors (TLRs) are a group of pattern recognition receptors and are implicated in the innate immunity against exogenous or endogenous dangerous ligands [28]. Importantly, TLR signalling has been indicated to be active in IL-1/HMGB1-promoted inflammation [29]. In particular, TLRs, such as TLR-2 and TLR-4 recognized HMGB1 and mediated the HMGB1-induced cytokine release [30].

In the present study, we investigated the mediator role of IL-1β and HMGB1 in the inflammation in disc annulus fibrosus cells. In particular, we examined the additive effect of both cytokines in disc annulus cells in the production of such cytokines as prostaglandin E2 (PGE2), IL-6, IL-8 and tumour necrosis factor alpha (TNF-α) [31–33], which are promoted in intervertebral disc degeneration. In addition, we examined the possible involvement of TLRs, receptors for advanced glycation endproducts (RAGE) and nuclear factor kappa-light-chain-enhancer of activated B-cells (NF-κB) signalling in such additive effect between IL-1β and HMGB1.

The article "IL-1β/HMGB1 signalling promotes the inflammatory cytokines release via TLR signalling in human intervertebral disc cells" was retracted in 2026. Reasons: manipulated data; manipulated images; plagiarized data; overlap with other authors' work.

## MATERIALS AND METHODS

### Cells and reagents

Human annulus fibrosus cells (HAFC, Cat. No. 4810) were pur-chased from the ScienCell Research Laboratories and were cultured under 5% CO_2_ at 37°C in nucleus pulposus cell medium (NPCM, Cat. No. 4801) (ScienCell Research Laboratories), which were supplemented with 10% fetal bovine serum (FBS) (Invitrogen), 100 units/ml penicillin and 100 μg/ml streptomycin (Sigma–Aldrich). Human recombinant IL-1β (BD Biosciences) and human recombinant HMGB1 (Abnova) were dissolved in NPCM with 2% FBS. A final concentration of 0, 0.5, 1, 2 or 5 ng/ml IL-1β or a final concentration of 0, 20, 40 or 80 ng/ml HMGB1 was utilized to treat 85%-confluent HAFC for 0, 6, 12, 24 or 48 h. Then HAFC were collected with a cell scratcher in ice-cold 1x PBS, and the cellular supernatant of treated cells was collected for the cytokine assay.

### ELISA analysis for supernatant levels of PGE2, TNF-α, IL-6 or IL-8

The supernatant levels of PGE2, TNF-α, IL-6 or IL-8 were quantified with the ELISA kit for each cytokine (Excellbio) according to each kit's guidance. Firstly, 100 μl serially-diluted standard samples or supernatant samples were added into the microplate and were incubated at 37°C for 1 h. Secondly, the plate was updated with 100 μl 1x antibody solution against PGE2, TNF-α, IL-6 or IL-8 in each well and was incubated 37°C for another 1 h. Thirdly, the plate was updated with 100 μl horseradish peroxidase-linked secondary antibody for incubation at 37°C for 30 min. Four time-washing was performed in each well of the plate with 100 μl PBS with Tween 20 (PBST) before incubation. Finally, the plate was inoculated with 100 μl substrate at dark for 15 min; the specific binding optical density was assayed immediately at 450 nm with a spectrophotometer (Bio-Rad Laboratories).

### Real-time quantitative PCR analysis

Total RNA was extracted from HAFC with TRIzol reagent (Life Technologies), was added with 1 μl SUPERase•In™ RNase Inhibitor (Thermo Scientific) and was assessed for quality by the OD260/OD280 ratio. Each RNA sample was quantified with One Step RT-PCT kit (Takara). And the RT-qPCR assay was performed for the reverse transcription firstly (at 42°C for 5 min, and then at 95°C for 10 s) and then for the PCR reaction (at 95°C for 5 s and at 60°C for 20 s, 40 cycles) using an ABI PRISM 7900HT Sequence Detection System (Applied Biosystems). The specificity of amplified products was determined by melting curve analysis. The relative expression levels of mRNA were calculated with the 2^−ΔΔCt^ method [34] and were presented as the relative quantitative value normalized to glyceraldehyde 3-phosphate dehydrogenase (GAPDH). The primers used in the study were as follows: MMP-1 forward (5′-gcc ttc caa ctc tgg agt aa-3′) and reverse (5′-ttg acc ctc aga gac ctt gg-3′); MMP-3 forward (5′- tgc caa aag atg ctg ttg att-3′) and reverse (5′-gag tca cct ctt ccc aga ct-3′); MMP-9 forward (5′-agc tgt att tgt tca agg atg-3′) and reverse (5′-aag ggg ccc tgc ggc cgg ctc-3′); tissue inhibitor of matrix metalloprotease-1 (TIMP-1) forward (5′-gtg ttt ccc tgt tta tcc atc-3′) and reverse (5′-cgt cca caa gca atg agt gc-3′); TLR-2 forward (5′-ttg tga ccg caa tgg tat ctg-3′) and reverse (5′-gcc ctg agg gaa tgg agt tta-3′); TLR-4 forward (5′-tgg tgt ccc agc act tca tc-3′) and reverse (5′-gcc agg tct gag caa tct cat a-3′); TLR-6 forward (5′-cca gga aaa agg gag act tct c-3′) and reverse (5′-tct aca atg ggg tgc aca gtg-3′); RAGE forward (5′-gag cca gaa ggt gga gca gta-3′) and reverse (5′-gca agg gca cac cat cct-3′); NF-κB forward (5′-tgc acc acc aac tgc tta gc-3′) and reverse (5′-tct tct ggg tgg cag tga tg-3′); IκBα forward (5′-acc tgg tgt cac tcc tgt tga-3′) and reverse (5′-ctg ctg ctg tat ccg ggt g-3′); GAPDH forward (5′-tgc acc acc aac tgc tta gc-3′) and reverse (5′-tct tct ggg tgg cag tga tg-3′).

The article "IL-1β/HMGB1 signalling promotes the inflammatory cytokines release via TLR signalling in human intervertebral disc cells" was retracted in 2026. Reasons: manipulated data; manipulated images; plagiarized data; overlap with other authors' work.

### Western blotting assay

Cytosol and nuclear section of proteins were prepared with the NE-PER™ Nuclear and Cytoplasmic Extraction Reagents (Thermo Scientific) in accordance with the manufacturer's protocols, and were quantified by the BCA Protein Assay Reagent Kit (Pierce). Equal amounts (30 μg) of samples were separated by SDS/12% PAGE and then were electrotransferred to nitrocellulose membrane (Millipore). The membranes were blocked with 2% BSA (Sigma–Aldrich) in PBS (4°C overnight), and then were incubated for 2 h at room temperature with specific primary antibody, against MMP-1, -3, -9, TIMP-1 or GAPDH (all from Abcam), against NF-κB/p65 or IκBα (both from Cell Signaling Technology). Then membranes were incubated with horseradish peroxidase-conjugated anti-rabbit antibody (Jackson Immuno Research) for 1 h at room temperature and the blots were detected using Enhanced Chemiluminescence reagent (Amersham Pharmacia Biotech).The integral optical density (IOD) of target band was analysed with Gel-Pro Analyzer Software 4.0 (Media Cybernetics), and was presented as a relative level of target protein IOD / GAPDH IOD.

### Statistical analysis

Quantitative data were presented as mean ± S.E.M. and was analysed with Student *t* test or the one-way analysis of variance (ANOVA) followed by the Tukey–Kramer test. *P* values less than 0.05 were considered significantly. All statistics were performed using Prism (GraphPad Software, version 5).

The article "IL-1β/HMGB1 signalling promotes the inflammatory cytokines release via TLR signalling in human intervertebral disc cells" was retracted in 2026. Reasons: manipulated data; manipulated images; plagiarized data; overlap with other authors' work.

## RESULTS

### IL-1β and HMGB1 additively promotes the inflammatory cytokines release in human intervertebral disc cells

In order to evaluate whether IL-1β and HMGB1 contribute to the inflammatory process in the degenerative human intervertebral disc, we investigated the effect of IL-1β and HMGB1 on human intervertebral disc cells *in vitro*. Firstly, intervertebral disc cells were incubated with 0, 0.5, 1, 2 or 5 ng/ml recombinant IL-1β for 24 h, and then the secretion of PGE2, TNF-α, IL-6 and IL-8 was examined. As indicated in Figure 1(A), there was a significant promotion to the supernatant levels of PGE2 and TNF-α by the treatment with 2 or 5 ng/ml IL-1β (*P*<0.05 or *P*<0.001) in the intervertebral disc cells. And the supernatant levels of IL-6 and IL-8 were also up-regulated by at least 1 or 2 ng/ml IL-1β (*P*<0.05, *P*<0.01 or *P*<0.001, Figure 1B). Secondly, the HMGB1 treatment was performed with a concentration of 0, 20, 40 or 80 ng/ml for 24 h, and the secretion of above-mentioned cytokines was also examined. Figures 1(C) and 1(D) demonstrated that the supernatant levels of PGE2 and TNF-α were also markedly up-regulated by 40 or 80 ng/ml HMGB1 in the intervertebral disc cells (*P*<0.05 or *P*<0.01). And the treatment with 80 ng/ml HMGB1 also up-regulated the supernatant levels of IL-6 and IL-8 (*P*<0.05 respectively, Figure 1D).

**Figure 1:** Supernatant levels of PGE2, TNF-α, IL-6 and IL-8 in the disc annulus fibrosus cells which were treated with IL-1β or HMGB1 Disc annulus fibrosus cells were treated with 0, 0.5, 1, 2 or 5 ng/ml IL-1β or with 0, 20, 40 or 80 ng/ml HMGB1 for 24 h, then the supernatant levels of PGE2, TNF-α, IL-6 and IL-8 were examined with ELISA methods. (A and B) Supernatant levels of PGE2 and TNF-α (A) or IL-6 and IL-8 (B) in the IL-1β-treated disc annulus fibrosus cells. (C and D): Supernatant levels of PGE2 and TNF-α (C) or IL-6 and IL-8 (D) in the HMGB1-treated disc annulus fibrosus cells. Results are presented as mean ± S.E.M. for quartic independent experiments. P values were calculated by Student t test between two groups, post the ANOVA test for the homogeneity of variance. *P<0.05, **P<0.01, ***P<0.001 or ns: no significance.

To elucidate whether there was an additive effect between IL-1β and HMGB1 on such cytokine promotion, we then treated the cells with 2 ng/ml IL-1β or (and) 40 ng/ml HMGB1 for 6, 12, 24 or 48 h for the supernatant cytokine assay. As indicated in Figure 2(A), the PGE2 was promoted from 12 to 48 h post treatment for 2 ng/ml IL-1β and from 24 to 48 h post treatment for 40 ng/ml HMGB1. And such promotion was more significant when cells were treated with both agents (*P*<0.001, Figure 2A), indicating an additive effect. And the promotion to TNF-α, IL-6 or IL-8 was also more significant by the combined treatment with IL-1β and HMGB1 than the treatment with either IL-1β or HMGB1 (*P*<0.05, *P*<0.01 or *P*<0.001, Figures 2B and 2D). Therefore, IL-1β and HMGB1 additively promotes the inflammatory cytokines release in human intervertebral disc cells.

The article "IL-1β/HMGB1 signalling promotes the inflammatory cytokines release via TLR signalling in human intervertebral disc cells" was retracted in 2026. Reasons: manipulated data; manipulated images; plagiarized data; overlap with other authors' work.

**Figure 2:** Additive inductions by IL-1β and HMGB1 of PGE2, TNF-α, IL-6 and IL-8 in disc annulus fibrosus cells Disc annulus fibrosus cells were treated with 2 ng/ml IL-1β or (and) with 40 ng/ml HMGB1 for 0, 6, 12, 24 or 48 h, then the supernatant levels of PGE2 (**A**), TNF-α (**B**), IL-6 (**C**) and IL-8 (**D**) were examined with ELISA methods. Results are presented as mean ± S.E.M. for quartic independent experiments. *P* values were calculated by parametric ANOVA (Tukey–Kramer post hoc) test. *P<0.05, **P< 0.01, ***P<0.001 or ns: no significance.

### IL-1β and HMGB1 additively up-regulates the expression of MMPs in human intervertebral disc cells

We then examined the expression of MMPs in the intervertebral disc cells post the treatment with IL-1β or (and) HMGB1. Figure 3(A) demonstrated that the mRNA levels of MMP-1 and MMP-3 were markedly up-regulated by the treatment with IL-1β (2 ng/ml) (*P*<0.05 or *P*<0.01). And 40 ng/ml HMGB1 significantly up-regulated the mRNA levels of both MMPs, in the presence of 2 ng/ml IL-1β, though the 40 ng/ml HMGB1 along did not significantly regulate the mRNA levels of both MMPs (*P*<0.05 or *P*<0.01, Figure 3A). And such additive regulation by IL-1β and HMGB1 was also found on MMP-9 mRNA expression (*P*<0.05 or *P*<0.01, Figure 3B), but not on the mRNA expression of TIMP-1 (Figure 3B). In addition, the expression of these MMPs in protein levels was also investigated by western blotting assay. As indicated in Figure 3(C), the protein levels of MMP-1, MMP-3 and MMP-9 were also additively up-regulated by IL-1β and HMGB1.

**Figure 3:** Expression of MMPs in the IL-1β- or/and HMGB1-treated disc annulus fibrosus cells Disc annulus fibrosus cells were treated with 2 ng/ml IL-1β or (and) with 40 ng/ml HMGB1 for 12 h, then the relative mRNA levels of MMP-1 (**A**), -3 (**A**), -9 (**B**) or TIMP metallopeptidase inhibitor 1 (TIMP-1) (**B**) to Glyceraldehyde 3-phosphate dehydrogenase (GAPDH) were examined with real-time quantitative PCR (RT-qPCR) method; (**C**) western blotting assay for MMP-1, -3, -9 and TIMP-1 in protein levels in the IL-1β- or (and) HMGB1-treated disc annulus fibrosus cells. Results are presented as mean ± S.E.M. for quartic independent experiments. Parametric ANOVA (Tukey–Kramer post hoc) test was performed for statistical significance analysis. *P<0.05, **P<0.01 or ns: no significance.

The article "IL-1β/HMGB1 signalling promotes the inflammatory cytokines release via TLR signalling in human intervertebral disc cells" was retracted in 2026. Reasons: manipulated data; manipulated images; plagiarized data; overlap with other authors' work.

### Involvement of TLR-4 and RAGE in the IL-1β- and HMGB1-induced CK release in human intervertebral disc cells

TLR signalling has been indicated to be active in IL-1/HMGB1-promoted inflammation [29]. In order to deduce the signalling pathway in the IL-1/HMGB1-promoted inflammatory cytokines release in human intervertebral disc cells, we then examined the expression of TLRs in the IL-1β/HMGB1-treated intervertebral disc cells. It was indicated that the expression of both TLR-2 and TLR-4 were markedly up-regulated by 2 or 5 ng/ml IL-1β (*P*<0.05, *P*<0.01 or *P*<0.001, Figures 4A and 4B). However, the TLR-6 expression was not significantly regulated by the IL-1β treatment (Figure 4C). Figure 4(D) demonstrated that the RAGE mRNA level was also markedly up-regulated by 2 or 5 ng/ml IL-1β (*P*<0.05 respectively). In addition, we examined the expression of TLR-4 and RAGE in the intervertebral disc cells, post the treatment with 40 ng/ml HMGB1. As indicated in Figures 4(E) and 4(F), the mRNA levels of both receptors were also significantly up-regulated by the HMGB1 treatment (*P*<0.05 respectively). Moreover, there was also an additive effect in the TLR-4/RAGE promotion by IL-1β and HMGB1. The mRNA levels of both receptors were higher in the cells with combined treatment with IL-1β and HMGB1 (*P*<0.05 or *P*<0.01, Figures 4E and 4F). Therefore, both TLR4 and RAGE were additively promoted by IL-1β and HMGB1 in human intervertebral disc cells.

**Figure 4:** Expression of TLRs and RAGE in mRNA levels in the IL-1β- or/and HMGB1-treated disc annulus fibrosus cells Disc annulus fibrosus cells were treated with 0, 0.5, 1, 2 or 5 ng/ml IL-1β for 12 h, then the relative mRNA levels of TLR-2 (**A**), -4 (**B**), -6 (**C**) or RAGE (**D**) to GAPDH were examined with RT-qPCR method; (**E** and **F**) relative mRNA levels of TLR-2 and -4 (**E**), TLR-6 and RAGE (**F**) to GAPDH in the IL-1β- or (and) HMGB1-treated (for 12 h) disc annulus fibrosus cells. Results are presented as mean ± S.E.M. for quartic independent experiments. *P* values in A–D were calculated by the parametric ANOVA (Tukey–Kramer post hoc) test; and *P* value in E–F was calculated by Student *t* test. *P<0.05, **P<0.01, ***P<0.001 or ns: no significance.

In addition, we knocked down TLR-4 in the in human intervertebral disc cells, and re-evaluated the IL-1β- and HMGB1-promoted release of inflammatory cytokines. As indicated in Figures 5(A)–5(C), the expression of TLR-4 in both mRNA (Figure 5A) and protein (Figures 5B and 5C) levels was markedly reduced in the siRNA-TLR-4 groups (*P*<0.01 or *P*<0.001, 30 or 60 nM). Figure 5(D) indicated that the promoted PGE2 release by both IL-1β (5 ng/ml) and HMGB1 (80 ng/ml) was significantly inhibited by the transfection with 60 nM siRNA-TLR-4 (*P*<0.05 or *P*<0.01). In addition, the IL-1β- and HMGB1-promoted release of TNF-α (*P*<0.05 or *P*<0.01, Figure 5E) and IL-6 (*P*<0.05 respectively, Figure 5F) was also reduced in the siRNA-TLR-4 groups. However, such inhibition was not significant for IL-8.

The article "IL-1β/HMGB1 signalling promotes the inflammatory cytokines release via TLR signalling in human intervertebral disc cells" was retracted in 2026. Reasons: manipulated data; manipulated images; plagiarized data; overlap with other authors' work.

**Figure 5:** siRNA-mediated TLR-4 knockdown inhibited the IL-1β- and HMGB1-induced CK release (**A**) TLR-4 mRNA level in the disc annulus fibrosus cells, which were transfected with 30 or 60 nM siRNA-Control or siRNA-TLR-4 for 24 h; (**B** and **C**) Western blot analysis of TLR-4 in protein level in the siRNA-Control- or siRNA-TLR-4-transfected disc annulus fibrosus cells for 24 h; (**D**–**G**) Supernatant levels of PGE2 (**D**), TNF-α (**E**), IL-6 (**F**) or IL-8 (**G**) in the IL-1β- (5 ng/ml for 24 h) or HMGB1- (80 ng/ml for 24 h) treated disc annulus fibrosus cells. Results are presented as mean ± S.E.M. for quartic independent experiments. *P* values were calculated by Student *t* test between two groups, post the ANOVA test for the homogeneity of variance. *P<0.05, **P<0.01 or ns: no significance.

### NF-κB signalling was additively promoted by IL-1β and HMGB1 in human intervertebral disc cells

NF-κB signalling pathway has been indicated to involve in the IL-1β-mediated inflammatory response in osteoblast cells [35] and to be activated by HMGB1 by various types of cells [36,37]. To further identify the signalling pathway underlining IL-1β/HMGB1-promoted inflammatory cytokines release in human intervertebral disc cells, we then examined the activation of NF-κB signalling in the intervertebral disc cells post IL-1β/HMGB1 treatment. Figure 6(A) demonstrated that there was a significantly high NF-κB/p65 mRNA level in the IL-1β-treated or HMGB1-treated intervertebral disc cells (*P*<0.05 or *P*<0.01); whereas the IκBα mRNA was markedly reduced by the 40 ng/ml HMGB1 (*P*<0.05). Moreover, the NF-κB/p65 mRNA up-regulation and the IκBα mRNA reduction were additively influenced by the treatment with both agents (2 ng/ml IL-1β and 40 ng/ml HMGB1) (*P*<0.05 or *P*<0.01). We then performed western blotting assay to evaluate the protein levels of NF-κB/p65 and IκBα in the IL-1β/HMGB1-treated intervertebral disc cells. As indicated in Figure 6(B), NF-κB/p65 protein level was also up-regulated by 2 ng/ml IL-1β or 40 ng/ml HMGB1 (*P*<0.05 respectively), and such up-regulation was more significant by the combined treatment with both agents (*P*<0.05 or *P*<0.01, Figure 6C). And the IκBα reduction was also recognized in protein level in the IL-1β- or HMGB1-treated intervertebral disc cells, particularly, such reduction was also additive (*P*<0.05 respectively). These data indicated that IL-1β and HMGB1 additively activated the NF-κB signalling pathway in intervertebral disc cells.

The article "IL-1β/HMGB1 signalling promotes the inflammatory cytokines release via TLR signalling in human intervertebral disc cells" was retracted in 2026. Reasons: manipulated data; manipulated images; plagiarized data; overlap with other authors' work.

**Figure 6:** Regulation on NF-κB/p65 and IκBα by IL-1β and HMGB1 in disc annulus fibrosus cells (**A**) Disc annulus fibrosus cells were treated with 2 ng/ml IL-1β or (and) with 40 ng/ml HMGB1 for 12 h, then the relative mRNA levels of NF-κB/p65 and IκBα to GAPDH were examined with RT-qPCR method. (**B** and **C**) Western blotting assay for (**B**) and relative levels of (**C**) NF-κB/p65 and IκBα in the disc annulus fibrosus cells, which were treated with 2 ng/ml IL-1β or (and) with 40 ng/ml HMGB1 for 24 h, with GAPDH as control; Student *t* test was performed for statistical significance analysis. *P<0.05, **P<0.01 or ns: no significance.

## DISCUSSION

IL-1β is one member of IL-1 family, which is closely linked to innate inflammatory and immune responses [11]. And IL-1β is thought to be one of the most strong proinflammation stimulator, promoting the production of multiple proinflammatory mediators such as cytokines, chemokines and MMPs [12–14]. Particularly, IL-1β is indicated to involve in the multiple pathological processes of intervertebral disc degeneration [16]. HMGB1 has been observed to mediate inflammation in multiple injury models [23–25]. Recently, HMGB1 has also been recognized as a potent proinflammatory mediator in degenerated human discs [26]. In the present study, we found that either IL-1β or HMGB1 promoted the inflammatory cytokines release in human intervertebral disc cells, the secretion of PGE2, TNF-α, IL-6 and IL-8 was significantly up-regulated in the supernatant of the intervertebral disc cells post the IL-1β or HMGB1 treatment. And the expression of MMP-1, -3 and -9 in both mRNA and protein levels in the intervertebral disc cells was also up-regulated by the treatment with IL-1β or with HMGB1. Furthermore, there was an additive effect between IL-1β and HMGB1 on such cytokine and MMP promotion. The combined treatment with IL-1β and HMGB1 exerted more significant promotion to PGE2, TNF-α, IL-6 and IL-8. And MMP-1, MMP-3 and MMP-9 in both mRNA and protein levels were also additively up-regulated by both mediators.

Both TLRs and HMGB1 are expressed in isolated human intervertebral disc cells and in native intervertebral disc tissue [38,39]. The present study for the first time indicated that IL-1β and HMGB1 additively promoted the expression of TLR-2, TLR-4 and RAGE, which is another HMGB1 receptor [40] in human intervertebral disc cells. It has been reported that the initiation of TLR signalling can cause the activation of NF-κB, and then result in the increased expression of proinflammatory cytokines such as IL-1, IL-6, IL-8 and TNF-α or MMPs in intervertebral discs [41]. We in the present study recognized the mediation of TLR-4 in the IL-1β- and HMGB1-induced CK release in human intervertebral disc cells. And the activation of NF-κB signalling was confirmed in the IL-1β/HMGB1-mediated additive promotion to inflammatory cytokines in intervertebral disc cells.

The article "IL-1β/HMGB1 signalling promotes the inflammatory cytokines release via TLR signalling in human intervertebral disc cells" was retracted in 2026. Reasons: manipulated data; manipulated images; plagiarized data; overlap with other authors' work.

Up to now, various types of cytokines have been recognized to be implicated and to contribute to the progression of IDD. However, it is not clear whether there is interplay among these cytokines in such process. The present study for the firstly time recognized such kind of interplay between IL-1β and HMGB1 in intervertebral disc cells. The additive promotion by IL-1β and HMGB1 to inflammatory cytokines might aggravate the progression of IDD.

## CONCLUSION

In summary, our study demonstrated that IL-1β and HMGB1 additively promotes the release of inflammatory cytokines and the expression of MMPs in human intervertebral disc cells. The receptors such as TLRs and RAGE and the NF-κB signalling were also additively promoted by IL-1β and HMGB1. Our study implied that the additive promotion by IL-1β and HMGB1 to inflammatory cytokines and MMPs might aggravate the progression of IDD.

## Abbreviations

ECM: extracellular matrix
FBS: fetal bovine serum
HAFC: human annulus fibrosus cells
HMGB1: high mobility group box 1
IDD: intervertebral disc degeneration
IL: interleukin
IOD: integral optical density
IVD: intervertebral disc
MMP: matrix metalloproteinase
RAGE: receptors for advanced glycation endproducts
TIMP-1: tissue inhibitor of matrix metalloprotease-1
TLR: toll-like receptor
TNF-α: tumour necrosis factor α

## References

[1] Urban J.P., Roberts S. (2003). Degeneration of the intervertebral disc. Arthritis. Res. Ther..

[2] Katz J.N. (2006). Lumbar disc disorders and low-back pain: socioeconomic factors and consequences. J. Bone Joint Surg. Am..

[3] Lotz J.C., Chin J.R. (2000). Intervertebral disc cell death is dependent on the magnitude and duration of spinal loading. Spine (Phila Pa 1976).

[4] Sambrook P.N., MacGregor A.J., Spector T.D. (1999). Genetic influences on cervical and lumbar disc degeneration: a magnetic resonance imaging study in twins. Arthritis. Rheum..

[5] Deyo R.A., Bass J.E. (1989). Lifestyle and low-back pain. The influence of smoking and obesity. Spine (Phila Pa 1976).

[6] Wang S.Z., Rui Y.F., Tan Q., Wang C. (2013). Enhancing intervertebral disc repair and regeneration through biology: platelet-rich plasma as an alternative strategy. Arthritis. Res. Ther..

The article "IL-1β/HMGB1 signalling promotes the inflammatory cytokines release via TLR signalling in human intervertebral disc cells" was retracted in 2026. Reasons: manipulated data; manipulated images; plagiarized data; overlap with other authors' work.

[7] Adams M.A., Roughley P.J. (2006). What is intervertebral disc degeneration, and what causes it?. Spine (Phila Pa 1976).

[8] Acaroglu E.R., Iatridis J.C., Setton L.A., Foster R.J., Mow V.C., Weidenbaum M. (1995). Degeneration and aging affect the tensile behavior of human lumbar annulus fibrosus. Spine (Phila Pa 1976).

[9] Lv F.J., Peng Y., Lim F.L., Sun Y., Lv M., Zhou L., Wang H., Zheng Z., Cheung K.M., Leung V.Y. (2016). Matrix metalloproteinase 12 is an indicator of intervertebral disc degeneration co-expressed with fibrotic markers. Osteoarthritis Cartilage..

[10] Aras A.B., Guven M., Balak N., Ayan E., Uyar S.B., Elmaci I. (2016). Evaluation of the association between matrix metalloproteinase 11 and intervertebral disc disease. Turk. Neurosurg..

[11] Dinarello C.A. (1994). The interleukin-1 family: 10 years of discovery. FASEB J..

[12] Dinarello C.A. (2011). Interleukin-1 in the pathogenesis and treatment of inflammatory diseases. Blood.

[13] Dinarello C.A. (2009). Immunological and inflammatory functions of the interleukin-1 family. Annu. Rev. Immunol..

[14] Zayed N., Afif H., Chabane N., Mfuna-Endam L., Benderdour M., Martel-Pelletier J., Pelletier J.P., Motiani R.K., Trebak M., Duval N., Fahmi H. (2008). Inhibition of interleukin-1beta-induced matrix metalloproteinases 1 and 13 production in human osteoarthritic chondrocytes by prostaglandin D2. Arthritis Rheum..

[15] Burke J.G., Watson R.W., McCormack D., Dowling F.E., Walsh M.G., Fitzpatrick J.M. (2002). Intervertebral discs which cause low back pain secrete high levels of proinflammatory mediators. J. Bone Joint. Surg. Br..

[16] Risbud M.V., Shapiro I.M. (2014). Role of cytokines in intervertebral disc degeneration: pain and disc content. Nat. Rev. Rheumatol..

[17] Genevay S., Finckh A., Mezin F., Tessitore E., Guerne P.A. (2009). Influence of cytokine inhibitors on concentration and activity of MMP-1 and MMP-3 in disc herniation. Arthritis Res. Ther..

[18] Le Maitre C.L., Hoyland J.A., Freemont A.J. (2007). Interleukin-1 receptor antagonist delivered directly and by gene therapy inhibits matrix degradation in the intact degenerate human intervertebral disc: an *in situ* zymographic and gene therapy study. Arthritis Res. Ther..

[19] Klune J.R., Dhupar R., Cardinal J., Billiar T.R., Tsung A. (2008). HMGB1: endogenous danger signaling. Mol. Med..

[20] Bianchi M.E., Agresti A. (2005). HMG proteins: dynamic players in gene regulation and differentiation. Curr. Opin. Genet. Dev..

[21] Bell C.W., Jiang W., Reich C.R., Pisetsky D.S. (2006). The extracellular release of HMGB1 during apoptotic cell death. Am. J. Physiol. Cell Physiol..

[22] Landsman D., Bustin M. (1993). A signature for the HMG-1 box DNA-binding proteins. Bioessays.

The article "IL-1β/HMGB1 signalling promotes the inflammatory cytokines release via TLR signalling in human intervertebral disc cells" was retracted in 2026. Reasons: manipulated data; manipulated images; plagiarized data; overlap with other authors' work.

[23] Yang R., Harada T., Mollen K.P., Prince J.M., Levy R.M., Englert J.A., Gallowitsch-Puerta M., Yang L., Yang H., Tracey K.J. (2006). Anti-HMGB1 neutralizing antibody ameliorates gut barrier dysfunction and improves survival after hemorrhagic shock. Mol. Med..

[24] Tsung A., Sahai R., Tanaka H., Nakao A., Fink M.P., Lotze M.T., Yang H., Li J., Tracey K.J., Geller D.A., Billiar T.R. (2005). The nuclear factor HMGB1 mediates hepatic injury after murine liver ischemia-reperfusion. J. Exp. Med..

[25] Kim J.Y., Park J.S., Strassheim D., Douglas I., Diaz D.V.F., Asehnoune K., Mitra S., Kwak S.H., Yamada S., Maruyama I. (2005). HMGB1 contributes to the development of acute lung injury after hemorrhage. Am. J. Physiol. Lung Cell Mol. Physiol..

[26] Gruber H.E., Hoelscher G.L., Bethea S., Ingram J., Cox M., Hanley E.J. (2015). High-mobility group box-1 gene, a potent proinflammatory mediators, is upregulated in more degenerated human discs *in vivo* and its receptor upregulated by TNF-alpha exposure *in vitro*. Exp. Mol. Pathol..

[27] Rajan N.E., Bloom O., Maidhof R., Stetson N., Sherry B., Levine M., Chahine N.O. (2013). Toll-like receptor 4 (TLR4) expression and stimulation in a model of intervertebral disc inflammation and degeneration. Spine (Phila Pa 1976).

[28] Lasker M.V., Nair S.K. (2006). Intracellular TLR signaling: a structural perspective on human disease. J. Immunol..

[29] Maroso M., Balosso S., Ravizza T., Liu J., Bianchi M.E., Vezzani A. (2011). Interleukin-1 type 1 receptor/Toll-like receptor signalling in epilepsy: the importance of IL-1beta and high-mobility group box 1. J. Intern. Med..

[30] Yu M., Wang H., Ding A., Golenbock D.T., Latz E., Czura C.J., Fenton M.J., Tracey K.J., Yang H. (2006). HMGB1 signals through toll-like receptor (TLR) 4 and TLR2. Shock.

[31] Willems N., Tellegen A.R., Bergknut N., Creemers L.B., Wolfswinkel J., Freudigmann C., Benz K., Grinwis G.C., Tryfonidou M.A., Meij B.P. (2016). Inflammatory profiles in canine intervertebral disc degeneration. BMC Vet. Res..

[32] Walter B.A., Purmessur D., Likhitpanichkul M., Weinberg A., Cho S.K., Qureshi S.A., Hecht A.C., Iatridis J.C. (2015). Inflammatory kinetics and efficacy of anti-inflammatory treatments on human nucleus pulposus cells. Spine (Phila Pa 1976).

[33] Johnson Z.I., Schoepflin Z.R., Choi H., Shapiro I.M., Risbud M.V. (2015). Disc in flames: roles of TNF-alpha and IL-1beta in intervertebral disc degeneration. Eur. Cell Mater..

[34] Schmittgen T.D., Livak K.J. (2008). Analyzing real-time PCR data by the comparative C(T) method. Nat. Protoc..

[35] Granet C., Miossec P. (2004). Combination of the pro-inflammatory cytokines IL-1, TNF-alpha and IL-17 leads to enhanced expression and additional recruitment of AP-1 family members, Egr-1 and NF-kappaB in osteoblast-like cells. Cytokine.

The article "IL-1β/HMGB1 signalling promotes the inflammatory cytokines release via TLR signalling in human intervertebral disc cells" was retracted in 2026. Reasons: manipulated data; manipulated images; plagiarized data; overlap with other authors' work.

[36] Tan Y., Wang Q., She Y., Bi X., Zhao B. (2015). Ketamine reduces LPS-induced HMGB1 via activation of the Nrf2/HO-1 pathway and NF-kappaB suppression. J. Trauma Acute Care Surg..

[37] Yang X., Wang H., Zhang M., Liu J., Lv B., Chen F. (2015). HMGB1: a novel protein that induced platelets active and aggregation via Toll-like receptor-4, NF-kappaB and cGMP dependent mechanisms. Diagn. Pathol..

[38] Klawitter M., Hakozaki M., Kobayashi H., Krupkova O., Quero L., Ospelt C., Gay S., Hausmann O., Liebscher T., Meier U. (2014). Expression and regulation of toll-like receptors (TLRs) in human intervertebral disc cells. Eur. Spine J..

[39] Rajan N.E., Bloom O., Maidhof R., Stetson N., Sherry B., Levine M., Chahine N.O. (2013). Toll-like receptor 4 (TLR4) expression and stimulation in a model of intervertebral disc inflammation and degeneration. Spine (Phila Pa 1976).

[40] Sims G.P., Rowe D.C., Rietdijk S.T., Herbst R., Coyle A.J. (2010). HMGB1 and RAGE in inflammation and cancer. Annu. Rev. Immunol..

[41] Wuertz K., Vo N., Kletsas D., Boos N. (2012). Inflammatory and catabolic signalling in intervertebral discs: the roles of NF-kappaB and MAP kinases. Eur. Cell Mater..

